# Diffusion Tensor Imaging Observation of Frontal Lobe Multidirectional Transcranial Direct Current Stimulation in Stroke Patients with Memory Impairment

This article has been retracted.

**DOI:** 10.1155/2022/2545762

**Published:** 2022-03-26

**Authors:** Hualiu Hua, Baixiang Zhang, Xiuling Wang, Yixian He, Mengting Lai, Ninghua Chen, Juan Liu

**Affiliations:** ^1^Department of Rehabilitation, Longyan First Affiliated Hospital of Fujian Medical University, Longyan 364000, China; ^2^Department of Rehabilitation, Longyan First Hospital, Longyan 364000, China

## Abstract

Stroke is a group of diseases caused by the sudden rupture or blockage of blood vessels in the brain that prevent blood from flowing into the brain, resulting in brain tissue damage and dysfunction. Stroke has the characteristics of high morbidity, high disability, and high mortality. To investigate the effect of multidirectional transcranial direct current stimulation (tDCS) of the prefrontal lobe in stroke memory disorder. We evaluated 60 patients with poststroke memory impairment who underwent magnetic resonance diffusion tensor imaging (DTI) during their admission to our hospital between January 2018 and December 2020. The patients were divided into the prefrontal group (*n* = 15), dorsolateral group (*n* = 15), prefrontal + dorsolateral group (*n* = 15), and pseudostimulation group (*n* = 15). Assessments using the Rivermead Behavioral Memory Test (RBMT), Montreal Cognitive Assessment Scale (MoCA), Lovingston Occupational Therapy Cognitive Scale (LOTCA), and frontal lobe fractional anisotropy (FA) were performed before and after treatment. The RBMT, MoCA, and LOTCA scores in the prefrontal + dorsolateral group were significantly higher than those in the dorsolateral, prefrontal, and sham groups (all *P* < 0.05). The posttreatment FA value of the frontal lobe was significantly higher in the prefrontal + dorsolateral group than in the dorsolateral, prefrontal, and sham stimulation groups (all *P* < 0.05). The FA value of the frontal lobe was significantly lower in patients with severe memory impairment than in patients with mild-moderate memory impairment (*P* < 0.05). The area under the receiver operating characteristic curve was 0.801 (95% CI: 0.678–0.925, *P* < 0.05), and the optimal cut-off value was 0.34, with a sensitivity and specificity of 81.60% and 72.70%, respectively. Prefrontal lobe + dorsolateral tDCS is beneficial in the treatment of post-stroke memory impairment. The DTI FA value can be useful in determining the degree of memory impairment.

## 1. Introduction

Cerebral apoplexy, also known as stroke and cerebrovascular accident, is a group of diseases caused by the sudden rupture of blood vessels in the brain or the inability of blood to flow into the brain due to vascular obstruction, resulting in brain tissue damage and dysfunction. Importantly, cerebral apoplexy is associated with high morbidity, a high disability rate, and a high mortality rate [1]. Poststroke cognitive impairment, one of the common complications of stroke, refers to a series of syndromes that meet the diagnostic criteria for cognitive impairment within 6 months after the clinical occurrence of stroke [2]. These include memory impairment and visual dysfunction that place a heavy burden on patients, families, and society. Therefore, there is an urgent need to improve cognitive impairment after stroke.

Transcranial direct current stimulation (tDCS) has been widely used in recent years in the study of poststroke cognition and motor ability. tDCS can stimulate the cerebral cortex through the anode; change the potential difference between the inner and outer membranes of neurons; stimulate the excitement and discharge of nerve cells; regulate the cerebral cortex activity; and affect the corresponding sensory perception, motor, and cognitive behaviors [3, 4]. Magnetic resonance diffusion tensor imaging (DTI), the only imaging method that can evaluate nerve fiber bundles in vivo, can noninvasively examine white matter integrity [5]. It indirectly reflects cell integrity and the pathological state by measuring the Brownian motion of free water molecules.

Fractional anisotropy (FA) values in the infarct foci and ipsilateral frontal lobe are significantly lower than those in the corresponding parts of the contralateral side. In addition, FA values in the frontal lobe region of the brain more accurately reflect the recovery of neurocognitive function [6, 7], further confirming the clinical value of DTI.

This paper aimed to investigate the efficacy of multidirectional tDCS in the treatment of poststroke memory disorders using magnetic resonance DTI. Ultimately, we aimed to more accurately evaluate the therapeutic effect of tDCS and prognosis of stroke patients.

## 2. Materials and Methods

We evaluated 60 patients with poststroke memory disorders admitted to our hospital between January 2018 and December 2020. The inclusion criteria were as follows: (1) stroke diagnosis according to the guidelines for the prevention and treatment of cerebrovascular diseases in China [8]; (2) a Rivermead Behavioral Memory Test (RBMT) score of [9] ≤21; (3) stable condition and ability to cooperate with treatment; and (4) informed consent to participate from both patients and their families. The exclusion criteria were as follows: (1) Rancho Los Amigos cognitive function grade <VII; (2) with comorbid malignant tumor, blood disease, autoimmune disease, and other serious diseases; and (3) a history of mental illness. The patients were randomly divided for stimulation into the prefrontal lobe group (*n* = 15), the dorsolateral group (*n* = 15), the prefrontal lobe + dorsolateral group (*n* = 15), and the sham stimulation group (*n* = 15) using the random number table method. The patient characteristics by group are shown in Table 1. There were no significant differences among the four groups.

Memory was assessed using RBMT, and memory impairment was defined as an RBMT score of ≤21. Specifically, mild, moderate, and severe memory impairment were defined as RBMT scores of 17–21, 10–16, and 0–9, respectively. Cognitive function, including visual-spatial executive ability, naming, memory, attention, and orientation, was assessed using the Montreal Cognitive Assessment Scale (MoCA) [10]. The total MoCA score is 30, and the higher the score, the better the cognitive function. Cognitive function was also assessed using the Lovingston Occupational Therapy Cognitive Scale (LOTCA) [11], which includes orientation, visual perception, spatial perception, and motor use. The total LOTCA score is 115, and the higher the score, the better the cognitive function.

Magnetic resonance imaging (MRI) was performed using a GE Signa HDxt 1.5 T MR superconducting scanner with an 8-channel phase matrix head coil. During imaging, the patients were required to lie flat on the examination bed in the supine position and were instructed to use earplugs to reduce noise. The head was fixed with sponge pads to reduce movement, and the patients were instructed to breathe calmly and keep still. Conventional sequences include T1-weighted imaging (TR, 400 ms; TE, 10 ms), T2-weighted imaging (T2WI; TR = 3000 ms, TE = 80 ms), and FLAIR (TR = 3000 ms, TE = 120 ms). A single excitation plane echo imaging technique was used in DTI (TR = 7800 ms, TE = 100 ms, *b* value = 0 and 1000 s/mm^2^, diffusion gradient direction = 10).

For image postprocessing, the original DTI image was processed using GE's ADW 4.5 image postprocessing workstation FuncTool software. Pseudocolor maps of anisotropy coefficient (FA) were obtained after posttreatment, and regions of interest (ROI) in the infarcts and ipsilateral frontal lobes were mapped. The ROI included the farthest possible margin of the whole lesion and the frontal lobe, with an area of 80–100 mm^2^. Each area was measured three times, and the measurements were averaged. Ipsilateral CST was reconstructed with the frontal lobe as the seed point, and the relationship between lesions and CST was determined.

Measurement data were expressed as ($\bar{x}\pm s$) and compared among groups using the *F* test. Meanwhile, enumeration data were expressed as *n* (%) and compared using the *χ*^2^ test. The diagnostic value of tDCS was analyzed using the receiver operating characteristic (ROC) curve. The inspection level was *α* = 0.05. All statistical analyses were performed using SPSS 22.0.

## 3. Experimental Test

There were no significant differences in the pretreatment RBMT, MoCA, and LOTCA scores among the four groups (*P* > 0.05). However, the posttreatment RBMT, MoCA, and LOTCA scores were significantly higher in the prefrontal lobe and dorsolateral groups than in the dorsolateral, prefrontal, and sham groups (*P* < 0.05). The RBMT, MoCA, and LOTCA scores in the prefrontal lobe and dorsolateral groups were also significantly higher than those in the sham stimulation group, but the difference was not significant (*P* > 0.05).  Table 2 displays pre and posttreatment RBMT, MoCA, and LOTCA scores by group.

There were no significant differences in the pretreatment FA values among the four groups (*P* > 0.05). However, the posttreatment FA values were significantly higher in the prefrontal lobe + dorsolateral group than in the dorsolateral, prefrontal, and sham groups (*P* < 0.05). The FA values in the prefrontal lobe and dorsolateral groups were significantly higher than those in the sham stimulation group, but the difference was not significant (*P* > 0.05).  Table 3 shows pre and posttreatment FA values in the frontal lobe by group.

In total, 40 and 11 patients had mild-moderate and severe memory impairment, respectively. The FA value of the frontal lobe was significantly lower in patients with severe memory impairment than in patients with mild-moderate memory impairment (*P* < 0.05).  Table 4 shows the comparison of FA values in the frontal lobes of patients with different degrees of stroke memory impairment.

The area under the ROC curve was 0.801 (95% CI: 0.678–0.925, *P* < 0.05). The optimal cut-off value was 0.34, with a sensitivity and specificity of 81.60% and 72.70%, respectively.  Figure 1 shows ROC curve.

## 4. Data Statistics and Result Analysis

As a common disease in the elderly, ischemic stroke can lead to impaired limb function and cognitive decline. Cognitive decline not only affects the patient's quality of life but also limb function. As a noninvasive and low-intensity technique, tDCS uses a constant microcurrent to regulate nerve cell activity in the cerebral cortex. It can stimulate the cerebral cortex through anodes, change the potential difference between the inner and outer membranes of neurons, promote the excitement and discharge of nerve cells, and regulate the activity of the cerebral cortex, affecting the corresponding sensory perception, motor, and cognitive behavior [12–14].

Magnetic resonance DTI can be used for quantitative analysis of pathological changes such as myelination and axonal reduction in the white matter regions of patients with ischemic stroke, providing a new method for exploring neuropathological changes in cognitive decline at the acute stage in patients with ischemic stroke. Stroke results in cerebral cortex damage, leading to different degrees of cognitive dysfunction. Cognitive dysfunction after stroke is closely related to the size, location, and number of lesions [14, 15]. The prefrontal cortex and the anterior side form the frontal lobo-subcortical circuitry, which is closely related to information processing, memory, and executive function. Any damage to this circuitry can lead to cognitive impairment [16]. Most stroke patients have decreased memory function.

The RBMT is an important tool for evaluating patient memory. The MoCA scale, as a comprehensive cognitive function screening tool, has high sensitivity and specificity for the early detection of stroke patients [17]. LOTCA can comprehensively and carefully assess the cognitive level and prognosis of stroke patients, thus making it clinically useful. Therefore, the RBMT, MoCA, and LOTCA cognitive rating scales were used as evaluation indices in this paper. Our results showed that posttreatment RBMT, MoCA, and LOTCA scores were significantly higher in the prefrontal lobe + dorsolateral group than in the dorsolateral, prefrontal, and sham stimulation groups. Further, the RBMT, MoCA, and LOTCA scores were significantly higher in the prefrontal lobe + dorsolateral group than in the sham group. These results indicate that patients had damage in multiple cognitive fields before treatment. Importantly, they support that the cognitive function of stroke patients is significantly improved after tDCS treatment. tDCS positive stimulation of the prefrontal lobe helped improve orientation, motor use, thinking and operation, attention and concentration, and cognitive dysfunction to a certain extent.

The frontal lobe is one of the most advanced parts of the brain, regulating memory, executive ability, abstract thinking ability, emotion, and other cognitive activities. Accordingly, frontal lobe damage can lead to various cognitive dysfunctions. The prefrontal lobe is composed of rich intercortical and subcortical fiber interactions that participate in the regulation of many higher cognitive functions. In cognitive activities, the frontal lobe has a higher integration function. Disruption of subcortical fiber connections can lead to cognitive impairment specific to the frontal lobe and its associated brain areas. This view is consistent with the popular “disconnection syndrome” hypothesis that stipulates that the pathophysiological changes of amnestic mild cognitive impairment are related to the disorder of interactions between different neuronal systems [18].

Episodic memory disorder is a sensitive indicator for the diagnosis of early Alzheimer's disease. Imaging studies have shown that the frontal lobe is involved in working and episodic memories, and it may be damaged in the early stages of cognitive impairment. FA is a widely recognized quantitative parameter of DTI that can objectively and indirectly reflect the structural integrity of white matter fibers. FA, which refers to the ratio of the anisotropic part to the total value of the dispersion tensor, can reflect the proportion of anisotropic components in the entire dispersion tensor [19]. In this paper, the FA values in the prefrontal lobe and dorsolateral groups were significantly higher than those in the dorsolateral, prefrontal, and sham groups. FA values were also significantly higher in the prefrontal lobe and dorsolateral groups than those in the sham stimulation group. This indicates that positive tDCS stimulation of the frontal lobe can improve orientation, motor use, thinking and operation, attention and concentration, and cognitive function to a certain extent.

The FA value, which ranges from 0 to 1, reflects the overall dispersion degree of water molecules. A decrease in FA values indicates a change in demyelination and a decrease in axon number, axon diameter, and axon structure in fiber bundles [20–23]. In stroke, some areas of the white matter that govern different functions are altered, and thus, FA values can be used to predict cognitive and other functional impairments caused by certain neurological diseases [24]. In the current paper, the FA value in the frontal lobe was significantly lower in patients with severe memory impairment than in those with mild-moderate memory impairment, indicating a loose arrangement of brain tissue structure and associated fiber damage [25–27]. The fiber tracts in this part are responsible for the interhemispheric connection between the prefrontal syncortices and are related to information monitoring in working memory and active extraction of information from the posterior syncortices [28]. Therefore, it is speculated that the reduced cognitive function of patients is related to structural changes and damaged integrity of axons in the fiber tracts.

Previous white matter studies mostly used traditional semiquantitative MRI methods. In T2WI and T2-FLAIR sequences, white matter injury is present as high signal intensity. However, this method cannot show the ultrastructure of white matter and has low sensitivity and specificity [29]. As such, it cannot be used for the early diagnosis of cognitive disease. Meanwhile, DTI can display anatomical details that cannot be provided by traditional MRI [30]. It can also show the shape and direction of white matter fiber bundles in vivo at the three-dimensional level. In addition, FA maps can reflect the characteristics of white matter damage across lesion stages. For example, in the early stages of white matter fiber damage, FA maps only show localized damage. As lesions progress, the normal shape of the fiber bundles gradually disappears, and FA values decrease sharply.

This provides a new objective basis for the early diagnosis, course transformation, and curative effect evaluation of various diseases, including cerebral infarction. The severity of reduced FA values has been reported to indirectly indicate the degree of infarction lesions and impairment in cognitive function. Consistent findings were found in the current paper. FA values in the frontal lobe showed a significantly high area under the ROC curve, sensitivity, and specificity for predicting severe memory impairment. These results support that FA values in the frontal lobe have significant value for diagnosing severe memory disorders.

## 5. Conclusion

In conclusion, prefrontal lobe + dorsolateral tDCS is beneficial in the treatment of poststroke memory impairment. The DTI FA value can be used to identify the degree of memory impairment.

This paper has some limitations. Further stratification, such as for site of disease, condition, and age, was not performed. In addition, the sample size was small owing to limited enrollment from time constraints. Lastly, the results have limited generalizability as xxx. Further large-scale clinical trials are needed to verify our findings.

## Figures and Tables

**Figure 1:** ROC curve.

**Table 1:** Clinicodemographic patient characteristics by group.

Groups	Cases	Sex		Age (years)	Course of disease (months)	Brain injury side		Types of stroke	
		Male	Female			Lift	Right	Cerebral infarction	Cerebral hemorrhage
Prefrontal lobe + dorsolateral group	15	9 (60.00)	6 (40.00)	66.65 ± 4.15	4.03 ± 0.98	4 (26.67)	11 (73.33)	9 (60.00)	6 (40.00)
Dorsolateral group	15	10 (66.67)	5 (33.33)	65.26 ± 3.89	3.92 ± 1.00	5 (33.33)	10 (66.67)	11 (73.33)	4 (26.67)
Prefrontal group	15	8 (53.33)	7 (46.67)	66.10 ± 4.20	3.98 ± 0.89	6 (40.00)	9 (60.00)	10 (66.67)	5 (33.33)
Sham stimulation group	15	10 (66.67)	5 (33.33)	66.03 ± 5.03	4.00 ± 1.02	5 (33.33)	10 (66.67)	10 (66.67)	5 (33.33)
*F*		0.776		0.26	0.034	0.600		0.600	
*P*		0.855		0.854	0.991	0.896		0.896	

**Table 2:** Pre and posttreatment RBMT, MoCA, and LOTCA scores by group.

Groups	Cases	RBMT		MoCA		LOTCA	
		Before treatment	After treatment	Before treatment	After treatment	Before treatment	After treatment
Prefrontal lobe + dorsolateral group	15	13.52 ± 1.89	18.03 ± 2.01abcd	23.15 ± 1.65	27.51 ± 1.57abcd	89.65 ± 6.03	103.36 ± 7.66abcd
Dorsolateral group	15	13.41 ± 2.03	16.60 ± 1.87ad	23.03 ± 1.73	25.26 ± 1.53ad	90.15 ± 5.97	95.59 ± 3.46ad
Prefrontal group	15	14.22 ± 1.94	16.15 ± 1.90ad	23.32 ± 1.82	25.10 ± 1.97ad	88.97 ± 7.10	96.03 ± 4.01ad
Sham stimulation group	15	13.98 ± 1.95	14.02 ± 1.91	23.19 ± 1.90	23.26 ± 1.88	89.24 ± 6.69	90.01 ± 5.57
*F*		0.574	11.171	0.068	14.87	0.095	15.282
*P*		0.634	0.000	0.977	0.000	0.963	0.000

Note: a, compared with the sham stimulation group, *P* < 0.05; b, compared with the prefrontal lobe group, *P* < 0.05; c, compared with the dorsolateral group (*P* < 0.05); d, compared with before treatment, *P* < 0.05.

**Table 3:** Pre and posttreatment FA values in the frontal lobe by group.

Groups	Cases	FA	
		Before treatment	After treatment
Prefrontal lobe + dorsolateral group	15	0.39 ± 0.10	0.65 ± 0.12abcd
Dorsolateral group	15	0.40 ± 0.08	0.51 ± 0.10ad
Prefrontal group	15	0.41 ± 0.07	0.50 ± 0.09ad
Sham stimulation group	15	0.38 ± 0.06	0.39 ± 0.07
*F*		0.402	18.222
*P*		0.752	0.000

Note: a, compared with sham stimulation group, *P* < 0.05; b, compared with prefrontal lobe group, *P* < 0.05; c, compared with dorsolateral group (*P* < 0.05); d, compared with before treatment, *P* < 0.05.

**Table 4:** Comparison of FA values in frontal lobe of patients with different degrees of stroke memory impairment.

Groups	Cases	FA	*t*	*P*
Mild to moderate	49	0.45 ± 0.09	3.105	0.003
Severe	11	0.36 ± 0.07		

## Data Availability

The simulation experiment data used to support the findings of this paper are available from the corresponding author upon request.
